# Cardiopulmonary Rehabilitation in Elderly Patients with Heart Failure: A Prospective Cohort Study

This article has been retracted.

**DOI:** 10.1155/2022/4923007

**Published:** 2022-04-01

**Authors:** Haitao Zhou, Aishu Dong, Xiaoqing Xu, Jianing Zhu, Bowen Shi

**Affiliations:** ^1^Department of Cardiology, The Second Affiliated Hospital and Yuying Children's Hospital, Wenzhou Medical University, Wenzhou 325000, Zhejiang, China; ^2^School of Nursing, Wenzhou Medical University, Wenzhou 325000, Zhejiang, China

## Abstract

**Objective:**

To determine the impact of cardiopulmonary rehabilitation administered through WeChat on exercising resilience and life quality in aged people with heart failure (HF).

**Methods:**

We conducted prospective cohort study that included 80 heart failure patients who were admitted to the Second Affiliated Hospital of Wenzhou Medical University from June 2018 to September 2020, 80 patients with heart failure. Patients were grouped according to their use of WeChat for rehabilitation. WeChat cohort provides remote supervision of rehabilitation and nursing guidance through WeChat. Specifically, the findings below were predetermined and compared across treatment groups utilizing analysis of variance corrected for baseline levels of the end measure and location: changes in the length of cardiopulmonary exercise tests, peak VO2, the proportion of predicted maximum VO2, and variation in the distance covered during the 6-minute walk distance (6MWD) assessment. Comparison of negative emotions between two groups, a Self-rating Depression Scale (SDS) and Self-rating Anxiety Scale (SAS), and Survey Short Form-36 (SF36) at baseline and at month 2.

**Results:**

In contrast with the control cohort, the WeChat cohort did not show any significant differences in general data (*P* > 0.05). After the rehabilitation, the WeChat group has a notably higher level in 6MWD than in the control group. Prior to the rehabilitation, there were no statistical gaps between the two cohorts in terms of SAS and SDS scores (*P* > 0.05). Even though the two cohorts saw a decline in SAS and SDS scores following nursing, the observation cohort indicated a much relatively low level in contrast with the control cohort (*P* < 0.05). The comparison of the SF-36 scores between the two cohorts revealed no significant differences (*P* > 0.05). Following nursing, the scores of the two cohorts declined significantly, with the control cohort scoring far lower than the other (*P* < 0.05).

**Conclusions:**

In summary, cardiopulmonary rehabilitation via WeChat is very beneficial for HF patients who are at a stable phase of the disease. It may substantially improve patients' exercise stamina, reduce adverse emotions, boost patients' quality of life, and have significant clinical relevance.

## 1. Introduction

Chronic heart failure (CHF) is a common clinical disease, which is the terminal stage of the development of a variety of heart diseases [1, 2]. The elderly is the population with a high incidence of chronic heart failure [3]. Due to the relatively poor immunity of the elderly, the body organs are in a state of continuous decline, so they have a high fatality rate [3, 4]. According to epidemiological investigation, the incidence of CHF in adults in developing countries is about 1%∼2% [5], and its incidence is proportional to age, and the prevalence of CHF in older people aged over 70 years is more than 10% [6]. Such a high incidence of CHF among the elderly, coupled with the elderly suffering from CHF physical decline, limited activities of daily living, easy recurrence of the disease, delayed course of the disease, and high rate of rehospitalization, has brought serious economic burden to the family and society. The rehabilitation goal of the CHF stable phase is to relieve symptoms and reduce the risk of future acute exacerbations. With the deepening of the health care concept, the use of appropriate nondrug rehabilitation has gradually become a hot topic in the management of the CHF stable phase [7, 8].

Cardiovascular and pulmonary rehabilitation (CVPR) is based on comprehensive evaluation and through the application of a variety of coordinated and targeted rehabilitations, including rehabilitation evaluation, exercise training, diet guidance, and health education, to improve the physiological and psychological state of patients [9, 10]. Unfortunately, engaging in physical activity is a common challenge in these chronic cardiopulmonary disease populations [11, 12]. Traditional center-based cardiopulmonary rehabilitation has been shown to improve outcomes. However, their utilization is extremely low, unavailable to the general population, and unsustainable [13]. Fewer than 13% of potential patients are referred by providers for pulmonary or cardiac rehabilitation while the incomplete rate is as high as 20% to 40% of patients referred [14]. In the case of a long distance from the site, inconvenient transportation, or the actual situation of the epidemic, internet-based methods can be adopted [15].

At present, WeChat is the most widely used smartphone application in China with a record of over 1 billion active monthly users [15]. Tele-rehabilitation allows for virtual treatment to be provided by permitting remote connections between patients and healthcare practitioners with the assistance of information and communication technologies [16]. WeChat, China's largest messaging platform, can send text, pictures, and videos [17, 18]. Instant messaging is possible [18]. Using WeChat, a unique approach to organizing and executing optimum care of HF patients may be feasible. We use WeChat remote rehabilitation to remotely supervise sports training. There are no relevant research reports on the topic of cardiopulmonary rehabilitation based on WeChat. Therefore, this study established a rehabilitation plan based on WeChat through a prospective cohort study, aiming to explore the enhancement in functional and quality-of-life outcomes.

## 2. Methods

### 2.1. Participants

We conducted the prospective cohort study that included 80 heart failure patients who were admitted to the Second Affiliated Hospital of Wenzhou Medical University from June 2018 to September 2020, 80 patients with heart failure. The following are the eligibility requirements: (1) heart failure patients (New York Heart Association functional classification III or IV), (2) age ≥65 years, (3) voluntary compliance with the study follow-up plan and ability to follow-up regularly, and (4) proficiency in the use of WeChat mobile apps. Patients who are capable of independently utilizing the fundamental operations of the WeChat software, including transmitting and receiving messages, initiating video calls, and reading articles. The following are the criteria for exclusion: (1) noncardiopulmonary comorbidities that restrict exercise (such as orthopedics and neuromuscular), (2) uncontrolled hypertension, (3) unstable HF, and (4) known serious mental illness (such as schizophrenia).

Approval for the present research was granted by the Ethics Committee of the Second Affiliated Hospital of Wenzhou Medical University, and all participants signed an informed consent form (LCKY2020-373).

### 2.2. Baseline Data Collection

The patients' clinical baseline data mainly included the following contents: (1) demographics: gender, age, smoking status, and body mass index (BMI); (2) complications: chronic renal failure, high blood pressure, chronic lung disease, diabetes, and hyperlipidemia; and (3) use of *β*-blockers and angiotensin-converting enzyme inhibitors/angiotensin receptor blockers (ACEI/ARB).

### 2.3. WeChat Group

Patients were grouped according to their use of WeChat for rehabilitation. The control cohort patients were treated with a standard regimen of medications and required hospital tests. At the time of the study, patients received educational guidance on maintaining a healthy lifestyle and were invited to engage in daily physical exercise. In WeChat group, the patients were provided with nursing intervention via WeChat In each session, nurses provided information on medication administration, physical activity, management of risk factors, smoking-quitting monitoring, nutritional consumption management, secondary prevention management, and other illnesses that may occur following CABG procedures. All courses are offered as short videos that are refreshed every week for a period of twelve months. Following the sending of each video lesson on the WeChat group, patients are asked to carefully review the video material and respond with the word “received” once they have completed the training. If patients have any questions concerning the video course, they can get in touch with the nurse via a WeChat group conversation or, if required, a face-to-face conversation with the nurse. It is the nurse's responsibility to respond to the patient's inquiries promptly and professionally. Moreover, in a case where the patients need clinical appointments, they can notify the nurse in the WeChat group, and the nurse will arrange an outpatient service. (2) Rehabilitation guidance: exercising is the foundation of rehabilitation recommendations, which included balance training, aerobic exercise, flexibility training, and weight training. Rehabilitation courses are also offered on a weekly basis in the manner of brief video sessions. We tracked the daily number of steps according to the results of patients' steps on WeChat and guided patients' family exercise according to the relevant results. Home workouts include 10–20 minutes of no-load ministrength exercise and 30 minutes of calisthenics three times and walking twice a week.

### 2.4. Outcome

The findings below were predetermined and compared across treatment groups utilizing analysis of variance corrected for baseline levels of the end measure and location: changes in the length of cardiopulmonary exercise tests, peak VO2, the proportion of predicted maximum VO2, and variation in the distance covered during the 6-minute walk distance (6MWD) assessment. Comparison of negative emotions between the quality of life in patients in the two cohorts, depression, and anxiety at baseline (M0) and at month 2 was performed. The Self-rating Depression Scale (SDS) [18] and Self-rating Anxiety Scale (SAS) [19] were utilized to evaluate depression and anxiety, respectively. The following are the SDS grading standards: ① <60: normal; ② 60∼69: mild depression; ③ 70∼79: moderate depression; and ④ ≥80 points: severe depression. SAS grading criteria are as follows: ① <60: normal; ② 60∼69: mild anxiety; ③ 70∼80 points: moderate anxiety; and ④ ≥ 80 points: severe anxiety. The Survey Short Form-36 (SF-36) [20] was employed to evaluate the overall quality of life. There are 36 items in total in the Italian version of the SF-36, which are organized into 8 categories: physical functionality, social functioning, role constraints due to physical difficulties, role restrictions associated with emotional issues, mental wellbeing, vitality, physiological discomfort, and overall health perceptions. Each category is given a score between 0 and 100, with 0 representing the worst health state and 100 representing the optimum health status. SF-36 scores were associated with superior self-perceived health. The assessment was conducted at the institute at a scheduled time. Investigators responsible for data collection were given specific training on measurement.

### 2.5. Statistical Analysis

This research is analyzed using the R software (Version4.00). All analyses are 2-tailed, *P* < 0.05 represents the difference. The measurement data are mean ± SD, and the counting data are displayed in percentage. The chi-square test or Student's *T*-test was utilized to assess the differences between the two cohorts.

## 3. Results

### 3.1. Subject Characteristics

The baseline characteristics of the cohort are presented in Table 1. No difference was observed in general data between the WeChat cohort and the Control cohort (*P* > 0.05).

### 3.2. Exercise Endurance

Before the rehabilitation, the 6MWD, peak oxygen consumption, and percentage of expected peak VO2, of these two cohorts showed no differences (*P* > 0.05, Table 2). Following the rehabilitation, the WeChat group has a considerably elevated level in 6MWD and peak oxygen consumption as opposed to the control cohort. The expected peak VO2 percentage change is not obvious.

### 3.3. Negative Emotions and Quality-of-Life Score

Before the rehabilitation, there were no obvious differences between the two cohorts in terms of SAS and SDS scores (*P* > 0.05). Even though the two cohorts saw a decline in SAS and SDS scores following nursing, the observation cohort indicated a much relatively low level in contrast with the control cohort (*P* < 0.05, Table 3). The comparison of the SF-36 scores between the two cohorts revealed no significant differences (*P* > 0.05). Following nursing, the scores of the two cohorts declined significantly, with the control cohort scoring far lower than the other (*P* < 0.05, Table 3).

## 4. Discussion

In the past, CHF patients were treated by lying down bed rest and limited physical activity can reduce the load on the heart [21]. With the modern heart rehabilitation [22] concept of the gradual development and treatment concept is constantly updated, more and more clinical guidelines are beginning to recommend exercise rehabilitation for patients with stable heart failure [23]. Heart failure is due to coronary heart diseases, hypertension, etc., that cause the systolic function and/or relaxation of the heart dysfunction occurs in a group of clinical syndromes, which are various cardiac syndromes [24, 25]. Severe manifestations or advanced stages of CHF, their mortality, and readmission rates have been high [24]. European Heart Association Acute and Chronic Heart 2016 Guidelines [26] for the diagnosing and treating of HF recommend that patients with chronic CHF should be actively carried out with cardiac rehabilitation based on exercise training. The benefit of exercise training for heart failure patients is motor energy increased strength, quality of life, and biomarkers [26].

Self-management of cardiac rehabilitation exercise is a part of the long-term treatment process of HF, and cardiac rehabilitation compliance is an important factor affecting cardiac rehabilitation. This study shows that in contrast with the control cohort, WeChat cohort education can substantially improve patients' compliance with cardiac rehabilitation exercise. First, WeChat group education is an organized, systematic, and targeted health education activity of the rehabilitation group, which can help patients acquire relevant knowledge of HF and improve their self-management level. Second, patients can communicate with each other in the WeChat group, which also helps patients realize the importance of rehabilitation exercises. Finally, WeChat can strengthen the monitoring of patients' compliance with rehabilitation, and rehabilitation exercise has a beneficial effect on the recovery of cardiac function, providing motivation for patients to adhere to cardiac rehabilitation exercise, so as to play a benign cycle.

The results of the current investigation showed that the SDS and SAS scores of the two cohorts reduced following the rehabilitation, with the observation cohort demonstrating a significantly lower level as opposed to the control cohort. According to this finding, cardiac rehabilitation nursing may dramatically attenuate negative emotions. We observed that the quality-of-life scores on symptoms, activities, and impact scores of the observation cohort were considerably elevated as opposed to those of the control cohort. It has also been suggested that the application of lung rehabilitation nursing might enhance the overall quality of life for those who are suffering from HF. Nevertheless, this investigation lacks a long-term follow-up, and cardiopulmonary rehabilitation therapies in patients with stable heart failure have been shown to reduce the course of the illness in certain cases. As a consequence, in the future, the sample size and the timeframe will be increased in order to obtain credible findings.

In conclusion, cardiopulmonary rehabilitation utilizing WeChat is very beneficial for CHF patients who are at a stable phase of the disease. It might significantly improve patients' exercise stamina, reduce adverse emotions, boost patients' quality of life, and have significant clinical relevance.

## Figures and Tables

**Table 1:** Baseline characteristics.

Characteristics	Control group	WeChat group	*P* value
*N*	40	40	
Age, years	68.0 ± 9.1	64.4 ± 12.6	0.147

*Sex, n (%)*			0.501
Male	23 (57.5)	20 (50.0)	
Female	17 (42.5)	20 (50.0)	
BMI, kg/m^2^	28.5 ± 4.6	28.9 ± 5.2	0.665

*History of smoking*			0.173
Yes	21 (52.5)	23 (57.5)	
No	19 (47.5)	17 (42.5)	

Left ventricular ejection fraction, %	35.0 ± 5.2	35.6 ± 5.2	0.590
*Previous medical history, n (%)*			
Myocardial infarction			0.544
Yes	23 (57.5)	26 (65.0)	
No	17 (42.5)	14 (35.0)	

*Hypertension*			0.617
Yes	30 (75.0)	28 (70.0)	
No	10 (25.0)	12 (30.0)	

*Hyperlipidemia*			0.115
Yes	14 (35.0)	21 (52.5)	
No	26 (65.0)	19 (47.5)	

*Diabetes*			0.356
Yes	23 (57.5)	27 (67.5)	
No	17 (42.5)	13 (32.5)	

*Stroke*			0.060
Yes	9 (22.5)	3 (7.5)	
No	31 (77.5)	37 (92.5)	

*Chronic kidney disease*			1.000
Yes	11 (27.5)	11 (27.5)	
No	29 (72.5)	29 (72.5)	

*Functional status by New York Heart Association Level*			0.083
I	12 (30.0)	5 (12.5)	
II	17 (42.5)	26 (65.0)	
III	11 (27.5)	9 (22.5)	

*Treatment, n (%)*			
*β*-Blocker	38 (95.0)	39 (97.5)	0.556
Angiotensin-converting enzyme inhibitors/angiotensin-receptor blockers	39 (97.5)	39 95.0)	0.556
Spironolactone	26 (65.0)	27 (67.5)	0.813

BMI: body mass index.

**Table 2:** Change from baseline to 8 weeks in outcomes.

	Control group	WeChat group	*P* value
6MWD, m			
0 week	308.4 ± 38.1	305.8 ± 56.4	0.889
8 week	346.2 ± 46.6	372.9 ± 45.2	0.012

*Peak oxygen consumption, mL/kg/min*			
0 week	16.2 ± 6.0	16.3 ± 5.2	0.679
8 week	16.9 ± 7.0	19.8 ± 5.0	0.008

*Percentage of expected peak VO2, %*			
0 week	53.2 ± 14.8	52.2 ± 14.0	0.916
8 week	53.8 ± 13.6	59.7 ± 17.4	0.102

6MWD: distance in 6-min walk test.

**Table 3:** Comparison of SAS, SDS and SF36 scores of two groups before and after rehabilitation.

	Control group	WeChat group	*P* value
*SAS score*			
0 week	71.5 ± 20.4	70.7 ± 20.5	0.840
8 week	69.8 ± 19.2	43.9 ± 18.1	<0.001

*SDS score*			
0 week	64.9 ± 9.0	66.7 ± 9.3	0.482
8 week	54.0 ± 13.7	44.7 ± 12.4	0.005

*SF36 score*			
0 week	87.2 ± 13.2	86.8 ± 10.2	0.513
8 week	87.9 ± 10.3	93.7 ± 10.7	0.005

SAS: Self-rating Anxiety Scales; SDS: Self-rating Depression Scale; SF36: Survey Short Form-36.

## Data Availability

The data used and/or analyzed during the current study are available from the corresponding author (Bowen Shi.) on reasonable request.
